The article "SLC8A1 antisense RNA 1 suppresses papillary thyroid cancer malignant progression via the FUS RNA binding protein (FUS)/NUMB like endocytic adaptor protein (Numbl) axis" was retracted in 2026. Reasons: concerns about the data; concerns about the results or conclusions.

# SLC8A1 antisense RNA 1 suppresses papillary thyroid cancer malignant progression via the FUS RNA binding protein (FUS)/NUMB like endocytic adaptor protein (Numbl) axis

**DOI:** 10.1080/21655979.2022.2073125

**Published:** 2022-05-21

**Authors:** Yunchao Xin, Xiaoling Shang, Xiaoran Sun, Guogang Xu, Yachao Liu, Yanbin Liu

**Affiliations:** a Department of Otolaryngology Head and Neck Surgery, the First Affiliated Hospital of Hebei North University, Zhangjiakou, Hebei, China; b Department of Gastroenterology, the First Affiliated Hospital of Hebei North University, Zhangjiakou, Hebei, China

**Keywords:** Papillary thyroid cancer, progression, lncRNA SLC8A1-AS1, FUS, Numbl

## Abstract

Papillary thyroid cancer (PTC) is one of the most prevalent endocrine malignancies and is associated with severe morbidity and high mortality. This study aimed to explore the role of long non-coding RNA (lncRNA) SLC8A1 antisense RNA 1 (SLC8A1-AS1) in the pathogenesis of PTC. In this study, we explored the function of SLC8A1-AS1 in PTC progression. We observed that the expression of SLC8A1-AS1 was downregulated in clinical PTC samples and PTC cell lines compared to that in normal controls. Cell counting kit (CCK)-8 assays demonstrated that the overexpression of SLC8A1-AS1 significantly reduced the proliferation of PTC cells. Consistently, apoptosis of PTC cells was enhanced by SLC8A1-AS1 overexpression. SLC8A1-AS1 overexpression attenuated the invasion and migration of PTC cells. Mechanistically, SLC8A1-AS1 maintained NUMB like endocytic adaptor protein (Numbl) mRNA stability by interacting with FUS RNA Binding Protein (FUS) in PTC cells. Depletion of Numbl reversed the inhibitory effect of SLC8A1-AS1 overexpression on PTC. Thus, we concluded that SLC8A1-AS1 suppresses PTC progression via the FUS/Numbl axis. Our findings provide novel insights into the mechanism underlying SLC8A1-AS1 attenuation of the malignant development of PTC, improving our understanding of the association between lncRNAs and PTC. SLC8A1-AS1 and FUS may be potential targets for PTC treatment.

## Highlights

- SLC8A1-AS is down-regulated in PTC samples.
- SLC8A1-AS overexpression reduces proliferation and induces apoptosis of PTC cells.
- SLC8A1-AS attenuates migration and invasion of PTC cells.
- SLC8A1-AS can inhibit Notch signaling in PTC cells.
- SLC8A1-AS maintains Numbl stability by interacting with FUS in PTC cells.

## Introduction

Thyroid cancer is a frequent endocrine malignancy characterized by a high death rate and growing incidence globally [1–3], and about 1% of tumor-associated morbidity is caused by thyroid cancer [4]. Moreover, four histological types of thyroid cancers have been reported: papillary, follicular, medullary, and poorly differentiated. Papillary thyroid cancer (PTC) is the most common histological subtype, accounting for 85–90% of all thyroid cancer cases. Despite the increasing rate of prognosis [5], aggressive metastasis in PTC cases still shows unsatisfactory outcomes [6]. Investigations of the mechanism of PTC development are crucial for the prognosis, therapy, and diagnosis of thyroid cancer patients [7,8]. Therefore, it is necessary to explore the mechanisms underlying PTC progression.

As a well-recognized type of non-coding RNA with a nucleotide length > 200, long non-coding RNAs (lncRNAs) play essential roles in cancer initiation and pathogenesis [9]. Several lncRNAs modulate thyroid cancer cells. For example, lncRNA XIST mediates thyroid cancer cell proliferation via miR-34a/MET/PI3K/AKT signaling [10]. The lncRNA MCM3AP-AS1 enhances the invasion and proliferation of thyroid cancer via modulating the miR-211-5p/SPARC axis [11]. Moreover, the lncRNA SLC8A1 antisense RNA 1 (SLC8A1-AS1) is abnormally expressed in oral squamous cell carcinoma [12]. Nevertheless, the role of lncRNA SLC8A1-AS1 in PTC remains unclear.

Importantly, lncRNAs can demonstrate their function by communicating with miRNAs or binding to RNA-binding proteins (RBPs) [13]. LncRNAs bind with RBPs to regulate target gene mRNA stability at the post-transcriptional level [13], and FUS RNA Binding Protein (FUS) is a critical mRNA stability modulator [14,15]. LncRNAs recruit FUS to enhance mRNA stability in human diseases [16,17]. However, as an mRNA stabilizer, the effect of FUS on PTC remains unclear. Moreover, Notch signaling has been identified as a crucial cellular pathway during PTC progression, in which NUMB like endocytic adaptor protein (Numbl) serves as an evolutionarily conserved factor and plays important roles in various processes such as targeting proteins for ubiquitination and endocytosis, asymmetric cell division, cell migration, and cell adhesion [18,19].

This study aimed to explore the role of SLC8A1-AS1 in PTC progression. Here, we revealed a crucial function of SLC8A1-AS1 in attenuating PTC tumourigenesis by maintaining Numbl stability through FUS recruitment.

## Materials and methods

### Cell culture and treatment

Normal human thyroid (Nthy-ori 3–1) and PTC (TPC-1 and B-CPAP) cell lines were purchased from Procell (Wuhan, China). The cells were cultured in a standard incubator at 37°C with 5% CO_2_ in RPMI-1640 (Gibco; Thermo Fisher Scientific, Waltham, MA, USA) with 10% fetal bovine serum (Gibco) and 1% penicillin/streptomycin [20]. The cells were treated with actinomycin D (2 μg/mL; Sigma-Aldrich, St. Louis, MO, USA) to analyze the mRNA stability. pcDNA3.1-SLC8A1-AS1, SLC8A1-AS1 small interfering (si) RNA, FUS siRNA, Numbl siRNA, and their corresponding negative controls (GenePharma, Shanghai, China) were transiently transfected into PTC cell lines using Lipofectamine 2000 (Invitrogen; Thermo Fisher Scientific, Inc.) at 37°C for 48 h, according to the manufacturer’s instructions.

### Cell counting kit-8 (CCK-8) assays

The cells were seeded in a 96-well plate (5 × 10^3^/well). CCK-8 reagent (10 μL, Dojindo, Japan) and 100 µL of phosphate-buffered saline (PBS) were added to each well for another 2 h at 37°C. The absorbance was recorded at 450 nm using a microplate reader (Bio-Rad, CA, USA) on days 1, 2, 3, and 4 [21,22].

### Transwell assays

For the Transwell assay, cells (1 × 10^5^) were seeded in fetal bovine serum (FBS)-free Dulbecco’s modified Eagle’s medium (DMEM) in the top chambers of a 24-well Transwell plate (Corning, USA), while complete DMEM was added to the lower chambers. After 24 h, the compartments were stained with 0.5% crystal violet and photographed under a microscope (Carl Zeiss, Jena, Germany). For the invasion assay, the top chambers were coated with Matrigel (Corning). Finally, 5–6 visual fields were selected under a microscope (Nikon, Japan) to count the number of migrated and invasive cells [23].

### Wound healing assay

A monolayer of TPC-1 and B-CPAP cells was formed after 24 h of incubation, reaching at least 80% confluency, and the monolayer was scraped using a 200 μL pipette. The cells were washed with PBS. Images of scratches were taken after 0 and 24 h using an inverted light microscope (Nikon, Japan) [24].

### Analysis of cell apoptosis

Cells (2 × 10^6^) were collected by binding buffer, and 5 μL propidium iodide (PI) and 5 μL AnnexinV-FITC (Beyotime Institute, Nantong, China) were plated in the samples for incubation for 15 min at 25°C. The results were analyzed using flow cytometry (BD Accuri C6 Plus, BD Biosciences, Franklin Lakes, NJ, USA) [25].

### RNA immunoprecipitation (RIP)

The RIP assay was conducted using the Magna RIP kit (Millipore, Germany) according to the manufacturer’s protocol. PTC cells were cross-linked by formaldehyde treatment for 10 min at 37°C. After washing with cold PBS, the cells were incubated in 4 mL cell lysis buffer for 15 min on ice. After nuclear extraction using a Dounce homogenizer (Wheaton; DWK Life Sciences), chromatin was sheared by sonication (25% power, 4.5 sec impact, 9 sec clearance, 14 times) at 37°C. PTC cells were then incubated with RIP buffer containing magnetic beads conjugated with anti-FUS or control antibodies (IgG) at 4°C for 6 h following DNase treatment for 30 min at room temperature. The beads were washed using the washing buffer, and the proteins were removed from the compounds via incubation with 0.1% SDS/0.5 mg/mL Proteinase K (30 min, 55°C). After washing, the RNA was extracted for qRT-PCR analysis [26].

### Quantitative PCR (qPCR)

Total RNA was isolated using TRIzol reagent (Invitrogen; Thermo Fisher Scientific, USA). cDNA was reverse-transcribed using the PrimeScript RT Master Mix (Takara, China). qRT-PCR was performed using SYBR Green (Takara, China) on the ABI PRISM® 7500 Sequence Detection System (Applied Biosystems, USA). GAPDH expression was used to normalize data, and the method of 2^−∆∆Ct^ was applied to calculate the results [27]. The primers used were as follows: Numbl 5′-TGACAGCATCAACGCTCTGT-3′, 5′-AGGCAGAAGTCCCTGTTGTG-3′; SLC8A1-AS1 5′-GCATATGTTGATGAGCAGGCA-3′, 5′-AGACTCAGTGACAGGGCTCA-3′; GAPDH 5′-CATGTTGCAACCGGGAAGGA-3′, 5′-GCCCAATACGACCAAATCAGAG-3′.

### Western blot analysis

Total protein was extracted using RIPA buffer (KeyGen, China). Protein concentration was quantified using a BCA protein kit (Beyotime, China). Proteins (30 µg) were separated by sodium dodecyl-sulfate polyacrylamide gel electrophoresis (SDS-PAGE) and transferred to polyvinylidene fluoride (PVDF) membranes (Millipore, USA). After blocking with 5% milk, membranes were incubated with primary antibodies overnight at 4°C, including Numb (ab155415, Abcam, USA), Numbl (ab37500, Abcam, USA), Notch1 (ab128076, Abcam, USA), Hes1 (ab71559, Abcam, USA), and β-actin (ab8227, Abcam, USA). Subsequently, the samples were incubated with secondary antibodies (Abcam, USA) for 1.5 h at room temperature and analyzed using enhanced chemiluminescence reagent (Beyotime, China) [28].

### Bioinformatics analyses

SLC8A1-AS1 expression profiles of GSE66783 and TCGA-PTC were obtained from the Gene Expression Omnibus (GEO) dataset website (https://www.ncbi.nlm.nih.gov/geo) and the Genomic Data Commons (https://portal.gdc.cancer.gov), respectively. Clinical information of PTC samples from The Cancer Genome Atlas (TCGA) datasets was obtained from supplementary data [29]. Survival analysis was performed using the Kaplan-Meier curve (K–M curve) method [30].

The relationships between SLC8A1-AS1, Numbl, and RBPs were predicted using the bioinformatics analysis tool Starbase v. 2.0 (http://starbase.sysu.edu.cn/index.php). The bioinformatics tool RPISeq (http://pridb.gdcb.iastate.edu/RPISeq) was used to predict the interaction probabilities of SLC8A1-AS1 and Numbl with FUS. For gene set enrichment analysis (GSEA), the Pearson correlation coefficient of other genes and SLC8A1-AS1 expression was calculated, and then the genes were sequenced according to the correlation coefficient. Gene sets were deposited in the GSEA Molecular Signatures Database (c2.cp.kegg.v7.1.symbols.gmt, https://www.gsea-msigdb.org/gsea/index.jsp).

### Statistical analysis

The results are expressed as mean ± SD. The Student’s *t*-test was used to compare the two groups. Differences between more than two groups were evaluated using one-way ANOVA followed by Tukey’s test. *P* < 0.05 indicated statistical significance.

## Results

This study aimed to explore the role of lncRNA SLC8A1-AS1 in the pathogenesis of PTC, which is still obscure. We explored the function of SLC8A1-AS1 in PTC progression. The expression of SLC8A1-AS1 was down-regulated in clinical PTC samples and PTC cell lines compared to normal controls. The overexpression of SLC8A1-AS1 significantly reduced PTC cell proliferation, and SLC8A1-AS1 maintains Numbl mRNA stability by interacting with FUS in PTC cells. Depletion of Numbl reversed the inhibitory effect of SLC8A1-AS1 overexpression on PTC.

### SLC8A1-AS is down-regulated in PTC samples

We detected SLC8A1-AS1 expression in clinical PTC samples from the TCGA database. SLC8A1-AS1 expression was lower in PTC samples than in normal samples (Figure 1(a)). Furthermore, with an increase in cancer stage, the expression of SLC8A1-AS1 decreased gradually, and the difference was significant (Figure 1(b)). In addition, in order to further verify the expression of SLC8A1-AS1 in PTC, we searched the GEO database and used the GSE66783 chip. It was found that the expression of SLC8A1-AS1 in PTC was also significantly decreased (Figure 1(c)). Moreover, the expression level of SLC8A1-AS1 had a significant effect on the disease-free interval (DFI) of PTC patients. Compared with the low SLC8A1-AS1 expression group, the DFI survival rate of PTC patients in the SLC8A1-AS1 high expression group was significantly higher (Figure 1(d)). Further Cox risk analysis found that with the increase in SLC8A1-AS1 expression, the patient’s risk of death decreased by 34.86% (Figure 1(e)), whereas other parameters (sex and age) were not risk factors. Consistently, the risk of death increased by 343.9% in phase III compared with phase I. Moreover, SLC8A1-AS1 expression was also decreased in PTC cells, with Nthy-ori 3–1 cells lines used as the control (Figure 1(f)).

**Figure 1.** SLC8A1-AS is down-regulated in PTC tissues and cell lines. (a) The expression of SLC8A1-AS1 in the clinical PTC samples (n = 272) and the normal samples (n = 48) from the TCGA database. (b) The expression of SLC8A1-AS1 in different stages of PTC from the TCGA database. (c) The expression of SLC8A1-AS1 in the PTC samples (n = 5) and the adjacent tissue samples (n = 5) from the GEO database (GSE66783). (d) Kaplan-Meier DFI survival plots in PTC patients from the TCGA database. (e) Cox risk analysis of PTC samples from the TCGA database. (f) The expression of SLC8A1-AS1 was measured by qPCR in the Nthy-ori 3–1, TPC-1, and B-CPAP cells. Data are presented as the mean ± SD of three independent measurements. ** *P* < 0.01, * *P* < 0.05.

### The overexpression of SLC8A1-AS reduces proliferation and induces apoptosis of PTC cells

The efficiency of SLC8A1-AS1 overexpression was validated in these cell lines (Figure 2(a)). SLC8A1-AS1 overexpression reduced the viability of TPC-1 and B-CPAP cells (Figure 2(b)). Moreover, apoptosis was induced in the SLC8A1-AS1-overexpressed cells (Figure 2(c)).

**Figure 2.** The overexpression of SLC8A1-AS reduces proliferation and induces apoptosis of PTC cells. (a) The expression of SLC8A1-AS1 was measured by qPCR. (b) The cell viability was analyzed by CCK-8 assays. (c) The cell apoptosis was measured by flow cytometry analysis. Data are presented as the mean ± SD of three independent measurements. ** *P* < 0.01.

### SLC8A1-AS attenuates migration and invasion of PTC cells

Wound healing assays showed that SLC8A1-AS1 overexpression inhibited wound healing (Figure 3(a)). Furthermore, overexpression of SLC8A1-AS1 significantly attenuated the invasion and migration of TPC-1 and B-CPAP cells (Figure 3(b)).

**Figure 3.** SLC8A1-AS attenuates invasion and migration of PTC cells. (a) The migration was assessed by wound healing assays. (b) The cell migration and invasion were analyzed by Transwell assays. Data are presented as the mean ± SD of three independent measurements. ** *P* < 0.01.

These results suggested that SLC8A1-AS1 decreased the migration and invasion of PTC cells.

### SLC8A1-AS can inhibit Notch signaling in PTC cells

Gene set enrichment analysis (GSEA) identified a potential association between SLC8A1-AS1 and Notch signaling (Figure 4(a)). As shown in Figure 4(b), Numb and Numbl inhibited the Notch pathway. Moreover, SLC8A1-AS1 overexpression enhanced the protein expression of Numb and Numbl and reduced the protein expression of Notch1 and Hes1 in TPC-1 and B-CPAP cells (Figure 4(c)), verifying that SLC8A1-AS1 inhibited Notch signaling in PTC cells. However, when pcDNA3.1-SLC8A1-AS1 and si-Fus were co-transfected into PTC cells, Notch1 and Hes1 protein expression increased and NUMBL protein expression decreased (Figure 4(c)).

**Figure 4.** SLC8A1-AS is able to inhibit Notch signaling in PTC cells. (a) The association of SLC8A1-AS1 with Notch signaling was identified in the GSEA using clusterProfiler R package. (b) Kyoto Encyclopedia of Genes and Genomes (KEGG) Pathway map of Notch signaling pathway. (c) The expression of Numb, Numbl, Notch1, and Hes1 was analyzed by western blot. Data are presented as the mean ± SD of three independent measurements. ** *P* < 0.01.

### SLC8A1-AS maintains Numbl stability by interacting with FUS in PTC cells

Next, we identified six overlapping RBPs interacting with SLC8A1-AS1 and Numbl mRNA and observed the potential binding probability of FUS with SLC8A1-AS1 and Numbl mRNA using bioinformatics analysis (Figure 5(a-c)). RIP assays showed that FUS interacted with SLC8A1-AS1 and Numbl in TPC-1 and B-CPAP cells (Figure 5(d,e)). Actinomycin D (ActD) mRNA stability analysis showed that SLC8A1-AS1 knockdown or FUS knockdown attenuated the stability of Numbl mRNA in TPC-1 and B-CPAP cells (Figure 5(f)), indicating that SLC8A1-AS1 maintains Numbl stability by interacting with FUS in PTC cells. Consistently, the ActD mRNA stability analysis showed that SLC8A1-AS1 overexpression promoted the mRNA stability of Numbl in TPC-1 and B-CPAP cells (Figure 5(g)), and FUS knockdown reversed this trend, indicating that SLC8A1-AS1 maintained Numbl stability by interacting with FUS in PTC cells.

**Figure 5.** SLC8A1-AS maintains Numbl stability by interacting with FUS in PTC cells. (a) The overlap analysis of the potential interacting RBPs with SLC8A1-AS1 and Numbl mRNA was performed using the starbase database. (b and c) The potential binding probability of SLC8A1-AS1 and Numbl mRNA with FUS was analyzed using the RPISeq database. (d and e) The interaction of FUS with SLC8A1-AS1 and Numbl was assessed by RIP assays in TPC-1 and B-CPAP cells. (f-g) The mRNA expression of Numbl was determined by qPCR assays in the cells. Data are presented as the mean ± SD of three independent measurements. ** *P* < 0.01.

### SLC8A1-AS attenuates malignant progression of PTC cells via regulating Numbl

We further validated the influence of the SLC8A1-AS1/Numbl axis on PTC development. Numbl siRNA was transfected into TPC-1 cells, and the depletion efficiency was validated by western blotting (Figure 6(a)). Overexpression of SLC8A1-AS1 increased the expression of Numbl. Numbl protein expression decreased after Numbl knockdown However, when PTC cells were co-transfected with pcDNA3.1-SLC8A1-AS1 and si-Numbl, Numbl protein expression was restored (Figure 6(b)). Interestingly, overexpression of SLC8A1-AS1 significantly repressed the viability of TPC-1 cells, and Numbl knockdown rescued this phenotype (Figure 6(c)). Moreover, Numbl knockdown notably reversed SLC8A1-AS1 overexpression-attenuated migration and invasion of TPC-1 cells (Figure 6(d)). Taken together, these data indicate that SLC8A1-AS1 reduces the malignant progression of PTC cells by regulating Numbl.

**Figure 6.** SLC8A1-AS attenuates malignant progression of PTC cells via regulating Numbl. (a-b) The protein expression of Numbl was examined by western blot. (c) The cell viability was analyzed by CCK-8 assays. (d) The cell migration and invasion were analyzed by Transwell assays. Data are presented as the mean ± SD of three independent measurements. ** *P* < 0.01.

## Discussion

PTC is a common endocrine neoplasm, and lncRNAs play crucial roles in PTC [11,31]. However, the influence of SLC8A1-AS1 on PTC progression remains unclear. SLC8A1-AS1 alleviates PTC malignant phenotypes by regulating FUS/Numbl signaling.

LncRNAs are known to participate in PTC progression. It has been shown that FOXD2-AS1 regulates PTC by mediating TERT levels via miR-7-5p [32]. Sara et al. reported a novel cerna regulatory mechanism with potential tumor suppressive activity through the klhl14/Pax8/BCL2/mir182-5p/mir20a-5p axis [33]. Lv reported that LINC0163 could regulate PTC progression via the inhibition of Wnt/β-catenin and activation of Axin2 [34]. Meanwhile, Liu found that lncRNA DUXAP8 could act as an oncogene in PTC, and these effects seem to be partly dependent on the miR-223-3p/CXCR4 axis [35]. Furthermore, previous studies have revealed that lncRNA SLC8A1-AS1 is involved in the development of various diseases, such as myocardial infarction and cancer. It has been reported that SLC8A1-AS1 relieves cardiac damage by activating cGMP-PKG signaling by repressing SLC8A1 in a myocardial infarction mouse model [36]. The lncRNA SLC8A1-AS1 serves as a biomarker for the early diagnosis of oral squamous cell carcinoma [12]. In this study, SLC8A1-AS1 expression was found to be reduced in PTC samples and cell lines. SLC8A1-AS reduced proliferation, invasion, and migration and enhanced apoptosis of PTC cells. This suggests that SLC8A1-AS is a novel tumor suppressor in PTC.

Notch signaling is a fundamental cellular process during malignant cancer progression and plays a key role in the initiation and development of PTC [37]. Moreover, targeting Notch signaling inhibits PTC progression and improves treatment effectiveness in PTC cases [37–39]. As a critical regulator of Notch signaling, Numbl has been found to decrease chemotherapy resistance, cancer stem cell-like properties, and tumourigenicity in breast cancer [40]. Moreover, FUS functions as an RBP of lncRNAs and has important impacts on cancer development [41]. Meanwhile, lncRNA DLX6-AS1 enhances invasion and migration by upregulating FUS and breast cancer [42]. In our mechanical exploration, we observed that SLC8A1-AS1 was able to inhibit Notch signaling in PTC cells. SLC8A1-AS1 maintained Numbl mRNA stability by interacting with FUS in PTC cells. SLC8A1-AS1 attenuates the malignant phenotype of PTC cells by regulating Numbl.

## Conclusions

In summary, we conclude that SLC8A1-AS1 suppressed the malignant progression of thyroid cancer via the FUS/Numbl axis. Our findings improve the understanding of the association between lncRNAs and PTC.

## Data Availability

The data used to support the findings of this study are available from the corresponding author upon reasonable request.
